The article "The Biomechanics Effect of Hamstring Flexibility on the Risk of Osgood-Schlatter Disease" was published in 2022. Journal: J Healthc Eng.

# The Biomechanics Effect of Hamstring Flexibility on the Risk of Osgood-Schlatter Disease

**DOI:** 10.1155/2022/3733218

**Published:** 2022-05-09

**Authors:** Xueying Zhang, Weiyan Ren, Yijie Duan, Jie Yao, Fang Pu

**Affiliations:** ^1^Key Laboratory of Human Motion Analysis and Rehabilitation Technology of the Ministry of Civil Affairs, Beijing Advanced Innovation Centre for Biomedical Engineering, School of Biological Science and Medical Engineering, Beihang University, No. 37 Xueyuan Road, Haidian District, Beijing 100191, China; ^2^State Key Laboratory of Virtual Reality Technology and System, Beihang University, No. 37 Xueyuan Road, Haidian District, Beijing 100191, China

## Abstract

**Background:**

The relationship between hamstring flexibility and the risk of OSD continues to be a debate, and whether hamstring stretching exercises should be considered as one of the conservative treatments of OSD is still unclear.

**Objectives:**

To investigate the relationship between hamstring flexibility and the risk of OSD by assessing the changes of loading on the tibial tuberosity caused by the changes of hamstring optimal lengths.

**Methods:**

Experimental data of a young adult running at 4 m/s were used, which were collected by an eight-camera motion capture system together with an instrumented treadmill. Muscle forces were estimated in OpenSim when hamstring optimal lengths changed in the range of 70–130% of the control case in 5% increments. The force and accumulated force of quadriceps muscle were calculated to evaluate the impact of hamstring optimal lengths on the loading on tibial tuberosity. The changes in muscle forces throughout the gait cycle were compared by using statistical parametric mapping (SPM). The average peak force and accumulated force of five gait cycles were compared.

**Results:**

Although the maximum force of the quadriceps muscle was slightly affected by changes in hamstring optimal lengths, the accumulated force of quadriceps muscle increased by 21.97% with hamstring optimal lengths decreased by 30% of the control case. The increase of the muscle force mainly occurred in the early stance phase and terminal swing phase (*P* < 0.05). However, when hamstring optimal lengths were longer than the control, it had a little effect on accumulated force of quadriceps muscle.

**Conclusions:**

The results of this study indicate that a shorter hamstring optimal length, which means lack of flexibility, can cause a high accumulated force on tibial tuberosity, thus increasing the risk of OSD. Hamstring stretching exercise is only effective for people with lack of hamstring flexibility.

## 1. Introduction

Osgood-Schlatter disease (OSD) is a traction apophysitis characterized by pain, swelling, and bony bump on the anterior aspect of the tibial tuberosity where the patellar tendon inserts into the bone [1, 2]. The prevalence of OSD is approximately 10% in adolescents, with 30% having bilateral symptoms [3], and it may be higher in those who are active in sports [4]. OSD generally appears in adolescents at the range of 8–14 in females and 10–15 in males [5]. It is commonly described as a self-limiting disease and resolves with closure of the tibial physis [3, 6]. However, teenagers with a history of OSD may not completely recover full joint functionality [7]. Therefore, effective interventions, such as stretching exercises, are often necessary to relieve the symptoms and speed up recovery.

It is widely accepted that OSD is a result of repeated contraction of the quadriceps muscle on the tibial tuberosity during the rapid growth stage of adolescents [4, 8]. Decreased quadriceps flexibility in OSD patients has been reported by some studies [9–11]. Close collaboration between the quadriceps and hamstring muscles, which are the agonist and antagonist muscles, can help to maintain joint stability during locomotion and other activities of daily living [12]. However, the relationship between hamstring flexibility and the risk of OSD is still unclear. Nakase et al. [13, 14] assessed the tightness of the hamstring muscles by measuring the straight leg raise (SLR) angle in a supine position and found that the SLR angle in OSD subjects was greater than that in the control group. Circi et al. [15], Kaneuchi et al. [16], and Ladenhauf et al. [2] also suggested that hamstring muscle tightness was one of the risk factors for OSD, and Ladenhauf et al. [2] pointed that physical therapy including hamstring stretching was essential and should be implemented in everyday practice routines for children who took part in regular sports activities. But other studies failed to find any relationship between them [4, 17]. Watanabe et al. [18] investigated pathogenic factors associated with OSD in adolescent male soccer players and reported that there was no significant difference in hamstring muscle tightness in comparison to the control group. Yanagisawa et al. [9] found that hamstring tightness did not increase with skeletal maturation. Therefore, it is uncertain whether hamstring flexibility affects the predisposition or the development of OSD.

Muscle optimal length is defined as the muscle length at which the force generated by muscle contractile elements is maximal [19]. Hamstring optimal lengths were significantly correlated with its flexibility score, the greater the flexibility score, the longer the hamstring optimal lengths [19]. Changing in the hamstring optimal lengths alters the length-tension curve and the joint range of motion [20–23], which may affect the capacity to produce force. Therefore, clarifying the effect of hamstring optimal lengths on the loading on the tibial tuberosity can help to understand the relationship between hamstring flexibility and the risk of OSD. This can also help to determine whether hamstring stretching, which is often used to improve hamstring flexibility, should be considered as one of the conservative treatments of OSD.

Accordingly, the aim of this study was to investigate the relationship between hamstring flexibility and the risk of OSD by assessing the changes of loading on the tibial tuberosity when the hamstring optimal lengths were altered based on OpenSim (Simbios, Stanford, CA, USA). We hypothesized that the loading on the tibial tuberosity increases when hamstring optimal lengths are reduced to a certain degree.

## 2. Methods

### 2.1. Experimental Data and Musculoskeletal Simulations

The experimental data used in the current study were from previously published studies by Hamner et al. and Rajagopal et al. [24, 25]. Briefly, the motion capture data and ground reaction forces of a 24-year-old male subject (height 1.78 m, mass 73 kg) running at 4 m/s were collected. A total of 54 infrared-reflecting markers were placed on the subject's body. The whole body kinematical data of the subject on the treadmill were recorded with an eight-camera optical motion capture system (Vicon, MX, Inc., Oxford, UK) at 100 Hz. Meanwhile, ground reaction forces were collected at 1000 Hz using an instrumented treadmill (Bertec, Inc., Columbus, Ohio, USA). Raw kinematic data and ground reaction forces were low-pass filtered using a zero-phase fourth-order Butterworth filter at the cutoff frequency of 15 Hz and critically damped filter.

A full-body musculoskeletal model called the Rajagopal model [25] (height 1.70 m, mass 75 kg) was used to perform the musculoskeletal simulations in OpenSim [26]. The model consisted of 80 musculotendon actuators (lower body) and 17 torque actuators (upper body) and had 20 degrees of freedom in the lower body, with three rotational and three translational degrees of freedom in the pelvis relative to the ground. The orientation of the femur (right and left) relative to the pelvis was described by the hip flexion angle, adduction angle, and rotation angle. The knee joint was simplified to only move through one degree of freedom. The ankle, subtalar, and metatarsophalangeal joints were modeled as pin joints with coordinates representing ankle dorsiflexion, ankle inversion, and toe flexion angles, respectively.

OSD is often reported in adolescents who frequently participate in sports [4, 15], and running is concluded in the majority of sports. Using a standard workflow (scale, inverse kinematics (IK), residual reduction algorithm (RRA), and computed muscle control (CMC)) in OpenSim, the generic model was scaled to the subject's anthropometry as determined during a static trial, and five running trials were used to perform the musculoskeletal simulations.

### 2.2. Changes in Hamstring Flexibility

Hamstring optimal lengths are defined as the hamstring muscle-tendon unit lengths at which maximal contraction forces are produced [21], and it has been investigated to significantly correlate to the flexibility score [19]. Furthermore, hamstring optimal lengths are difficult to measure in vivo. In the Rajagopal model, the optimal lengths were taken directly from the mean optimal fiber length measured by Ward et al. [27], who disassembled 27 muscles from 21 human lower extremities to characterize muscle fiber length. Therefore, the hamstring optimal lengths collected by Ward et al. [27] were used as the control in the current study. Given that the hamstring flexibility of some people maybe 30% less than that of the control group [28] and the hamstring muscles are composed of the biceps femoris long head (BF-lh), the biceps femoris short head (BF-sh), semimembranosus (SM), and semitendinosus (ST) [29], the optimal lengths of BF-lh, BF-sh, ST, and SM were progressively changed together in the range of 70–130% of the control case in 5% increments in the current study. Baseline simulations of five running gait cycles were conducted. Additional simulations were then created for each gait cycle at progressively changed of hamstring optimal lengths. All simulations tracked normal gait patterns when the hamstring optimal lengths changed.

### 2.3. Statistical Analysis

OSD is thought to be the result of repetitive high forces being transferred from the quadriceps muscle to the insertion of the patellar tendon on the tibial tuberosity [8]. In this research, the peak force and accumulated force of quadriceps muscle before and after hamstring optimal lengths changed were calculated, and the accumulated force was defined as the accumulation of quadriceps muscle force overtime of a gait cycle (∫ Force dt). To analyze the effect of the hamstring optimal lengths' changes on the quadriceps muscle force throughout the gait cycle, the paired statistical parametric mapping (SPM) *t*-tests [30, 31] were used from an open-source spm1d package (https://www.spm1d.org) [32] in MATLAB (R2019a, The Mathworks Inc., Natick, USA). A value of *P* < 0.05 was considered statistically significant for all tests. Data were presented as mean ± standard deviation for five running trials. Before statistical analysis, all data were tested for normal distribution with a Shapiro–Wilk test in IBM SPSS Statistics 25 (IBM Corporation, NY, USA).

## 3. Results

The results were verified by comparing the simulated muscle activity with the EMG data in Rajagopal's research [25] when hamstring optimal lengths were not changed, which showed that the timing of the simulated muscle activations was consistent with measured EMG signals in running. When simulations after changing the optimal lengths were carried out, the results for RRA and CMC were acceptable. Both root mean square of position errors (RMS pErr) and the maximum of position errors (MAX pErr) between the model kinematics and experimentally measured kinematics being less than 4° (or 2 cm for translations), which means the simulations reproduced the subject's movement well.

The accumulated force of quadriceps and hamstring muscles increased with the decrease of hamstring optimal lengths, and both hamstring and quadriceps muscles experience their maximum accumulated force when hamstring optimal lengths were reduced by 30% (Figure 1(a)). However, the accumulated force decreased slightly with the increase of hamstring optimal lengths.

The changes of hamstring optimal lengths had a little effect on the peak force of the quadriceps muscle. However, it had a greater impact on the peak force of hamstring muscles (Figure 1(b)). The maximum change of quadriceps peak force was 386.99 N, and for hamstring muscles, it reached 1263.87 N, both of which occurred when the optimal lengths reduced by 30%.

When hamstring optimal lengths were reduced by more than 20%, the accumulated force of the quadriceps muscle increased rapidly (Figure 2). A 30% reduction in hamstring optimal lengths caused the greatest change in accumulated force (increasing by 21.97%). But increased optimal lengths had a little effect on the accumulated force, and its change was only 1.07% when the optimal lengths increased by 30%.

The maximum change in peak force of quadriceps muscle was experienced when the hamstring optimal lengths were reduced by 30%, resulted in an increase in peak force of 387 N (an increase of 5.79%) than the control case, while the peak force changed by no more than 3% in all other cases (Figure 3).

When the hamstring optimal lengths were reduced by 20% from the control case, the quadriceps muscle force increased significantly in the loading response of the stance phase (*p*=0.017, Figure 4(a)). The significant increase of force occurred in the terminal swing phase when the length was reduced by 25% (Figure 4(b)). Further reducing the optimal lengths by 30% led to a significant increase in both loading response of the stance phase and the terminal swing phase (*P* < 0.001, Figure 4(c)). There was no significant difference in other cases.

## 4. Discussion

To the best of the authors' knowledge, no other studies have investigated the relationship between hamstring flexibility and the risk of OSD from the perspective of biomechanics. In this work, the influence of the hamstring optimal lengths on the loading on the tibial tuberosity, which was associated with quadriceps muscle force, was evaluated quantitatively. The major findings of the current study were that the accumulated force of quadriceps muscle increased significantly when the hamstring optimal lengths were shorter than the control case, the significant increase in accumulated force mainly occurred in the loading response of stance phase and the terminal swing phase of the gait cycle, and the force and accumulated force on quadriceps muscle was less effected by hamstring optimal length when it was greater than the control case. The results suggest that hamstring stretching exercises to improve hamstring flexibility will help reduce the risk of OSD, but only when the hamstring flexibility is poor.

The study found that the changes in the hamstring optimal lengths had little impact on the maximum force of the quadriceps muscle. Thelen et al. [33] reported that hamstring muscle-tendon lengthening begins at about 45% of the gait cycle and reaches its peak length at about 90% of the gait cycle during sprinting. EMG analysis showed that the hamstring muscles were more active in the last 20% of the gait cycle during sprinting [34, 35]. However, the quadriceps muscle force reaches its peak at around 14% of the gait cycle. At this phase, hamstring muscles were not as active as in the terminal swinging phase and predominantly performed concentric actions. Therefore, the changes of the hamstring optimal lengths had a little effect on its force (Figure 5(a)). As the knee joint was flexed and extended, the hamstring and quadriceps muscles acted as an agonist and antagonist, respectively, which helped to explain why there was only a minor variation in the peak force of the quadriceps muscle. This result indicates that the relationship between hamstring flexibility and the risk of OSD may not be illustrated by the peak force of the quadriceps muscle.

The significant increase of quadriceps muscle force mainly occurred in the loading response of the stance phase and the terminal swing phase when hamstring optimal lengths were 20% shorter than the control. During the terminal swing phase, the hip was flexed and the knee was extended. Hamstring muscles were highly active at this stage while predominantly performing eccentric actions, which extended from the terminal swing phase to the loading response of the stance phase [33]. The length-tension curve was on the descending limb, and the active force was decreasing while the passive force increased at this time [36]. Shorter hamstring optimal lengths, which meant lack of flexibility, caused greater passive force when hamstring muscles performed eccentric actions and then led to the increase of hamstring muscle force in the loading response of the stance phase and the terminal swing phase (Figure 5(a)). As the agonist and antagonist muscles, the coactivation mechanism of the quadriceps and hamstring was integral to the maintenance of knee joint stability during locomotion and other daily activities [12]. Therefore, the changes of quadriceps muscle force were mainly caused by the change of hamstring muscle force at those two stages (Figure 5(b)). Although quadriceps muscle force did not reach the maximum in the loading response of the stance phase and the terminal swing phase, the increased force was unfavorable to the development of the tibial tubercle. In addition, the cumulative effect of the increased quadriceps muscle force on the tibial tubercle should also be considered.

In the present study, the accumulated force of quadriceps muscle increased significantly when the hamstring optimal lengths were 20% or shorter than the control. OSD was caused by continued and repetitive loads placed upon the tibial tuberosity [3, 37, 38], and repetitive strain mainly comes from the pull of the quadriceps muscle [39, 40]. It indicated that more attention should be paid to the periodic accumulation of quadriceps muscle force when exploring the relationship between hamstring flexibility and the risk of OSD. Therefore, the accumulated force of the quadriceps muscle was used to describe the persistent loading on the tibial tuberosity in this study. Noteworthy, the increase of quadriceps muscle force in the loading response of the stance phase and the terminal swing phase was responsible for the significant increase of the accumulated force in this study. The result suggests that the early stance phase and terminal swing phase should be given more attention when performing conservative treatments for adolescents. To our knowledge, this continues the first study to explore the risk factors associated with OSD by using the accumulated force on tibial tuberosity, which may provide a new perspective for the study of OSD.

In conclusion, the current study offers some important insight into the conservative treatment of OSD. It will be of great importance to perform hamstring stretching exercises for people with lack of hamstring flexibility. However, hamstring stretching is ineffective in adolescents or OSD patients with normal or good hamstring flexibility. The results of the present study can help to understand why it is still unclear whether hamstring stretching exercises should be considered as one of conservative treatments of OSD according to previous literature. This is because the hamstring flexibility should be examined before making a decision. Hamstring flexibility can be evaluated using a standard physical therapy technique: the SLR test. The flexibility of hamstring is classiﬁed as tight (<60°), normal (60–90°), or loose (>90°) based on the SLR angle [28]. For adolescents in the high-risk age bracket for OSD (10–15 years in boys and 8–14 years in girls [5]), the SLR test should be performed regularly, and hamstring stretching exercises or other effective measures [41–43] should be taken once the hamstring flexibility is classiﬁed as tight. For OSD patients, other factors should be found, and corresponding treatment measures should be taken if the hamstring flexibility is classified as normal or loose.

There are some limitations to this study. First, all simulations were forced to a track normal pattern. However, normal gait cannot be maintained in adolescents whose hamstring muscles are shortened during running. It was compensated by changing the muscle force to maintain a normal gait in this study. Second, the parameters of the full-body musculoskeletal model used to perform simulations in this study, such as musculotendon parameters and skeletal structure, come from adults, which might not be fully representative of adolescents. The model whose parameters come from teenagers will be used in future research. Third, running was the only motion considered in this study, but future studies should consider expanding the scope to cover other motions and sports.

## 5. Conclusions

The results indicate that compared with the peak force of quadriceps muscle, accumulated force may be a better index reflecting the influence of changing hamstring optimal lengths on the loading on the tibial tuberosity. In this work, the significant increase of accumulated force is strongly associated with the increase of quadriceps muscle force in the loading response of the stance phase and the terminal swing phase when hamstring flexibility is poor, which indicates that more attention should be given to these two stages when training. The study further revealed that hamstring stretching exercises only work for people with lack of flexibility, and it is necessary to check the hamstring flexibility at first.

## Figures and Tables

**Figure 1:** The accumulated force (a) and peak force (b) of the quadriceps and hamstring muscles with changes in hamstring optimal lengths.

**Figure 2:** Variation in accumulated force of the quadriceps muscle with changes in hamstring optimal lengths.

**Figure 3:** Variation in peak force of quadriceps muscle with changes in the hamstring optimal lengths.

**Figure 4:** Force (A) and SPM{*t*} (B) curves. The force is described as mean (hard line) ± standard deviation (shaded area). The shaded areas on the SPM{*t*} curve show the track locations where the SPM{*t*} curve exceeded the critical threshold (dotted line). *P* values are provided for these suprathreshold clusters. (a) Optimal lengths reduced by 20%. (b) Optimal lengths reduced by 25%. (c) Optimal lengths reduced by 30%.

**Figure 5:** Changes in quadriceps muscle force (a) and hamstring muscle force (b) during a gait cycle. The force is described as mean (hard line) ± standard deviation (shaded area). The vertical axis represents the difference in muscle force from the model with unadjusted hamstring optimal lengths.

## Data Availability

The datasets used and/or analyzed during the current study are available from the corresponding author upon request.
